# Public Health Practitioners' Knowledge towards Nicotine and Other Cigarette Components on Various Human Diseases in Pakistan: A Contribution to Smoking Cessation Policies

**DOI:** 10.1155/2022/7909212

**Published:** 2022-10-03

**Authors:** Abdul Hameed, Daud Malik

**Affiliations:** Department of Research, Alternative Research Initiative (Pvt.) Ltd., Pakistan

## Abstract

Smoking cessation seems to be a weak link in the struggle against tobacco epidemic in Pakistan. Awareness regarding nicotine is lacking not only in the general population but also among public health practitioners. This lack of knowledge is one of the key barriers to bringing down the prevalence of smoking. Using primary survey data and nonparametric econometric techniques, this study assesses the knowledge of nicotine and harm reduction among public health practitioners in Pakistan. Results indicate physicians have misconceptions about nicotine. The majority of the medical professionals associate nicotine use with birth defects, cancer, cardiovascular illness, and chronic obstructive pulmonary disease (COPD). More than two-thirds of doctors (70%) strongly agreed and 17.9% somewhat agreed with the statement that nicotine causes cancer. This study suggests physicians need to be better informed about the fact that nicotine in tobacco products is addictive while chemicals, particularly those causing combustion, are the primary risk sources for tobacco-related illnesses. Misconceptions regarding nicotine can be quickly remedied with communication interventions. This study also suggests that alternative nicotine delivery systems can help smoking cessation and reduce the consumption of combustible tobacco in Pakistan.

## 1. Introduction

Tobacco pandemic kills more than eight million people every year. The majority of the world's 1.3 billion tobacco smokers reside in low- and middle-income nations “where the burden of smoking-related disease and mortality is greatest”. As a result, smoking plays a considerable role in health disparities [1, 2]. The use of tobacco and its effects on countries vary. The implementation of comprehensive tobacco control programs has led to decrease in smoking prevalence in the developed countries, while it has registered increase in the developing and low income countries. Since 1970s, cigarette smoking has decreased dramatically in the higher-income or developed nations, primarily due to growing public awareness about the importance of health, the construction of smoke-free indoor areas, and the introduction of control measures such as pricing, laws, and taxes [2]. However, population growth is contributing to an increase in the number of smokers globally [3].

In South Asia, smoking is the most common and one of the most important preventable causes of liver, oral and throat cancer, COPD, heart disease, and stroke. India, Bangladesh, and Pakistan are particularly vulnerable [4, 5]. Pakistan is one of 15 nations with a high burden of tobacco-related diseases. More than 23.9 million people (31.8% men and 5.8% women) use tobacco in various forms, including smoking and smokeless tobacco. However, 15.6 million people (22.2% men and 2.1% women) are active smokers, and 3.7 million smoke sheesha—a water-pipe composed of a head (filled with moist tobacco), a central stem going to a water bowl at the bottom, and a hose with a mouthpiece on the end [6]. The adult cigarette smoking and barriers to cessation have become one of the most critical issues in Pakistan. Moreover, lack of knowledge seems to be the major reason for not seeking medical assistance for quitting smoking. Knowledge about nicotine replacement therapy (NRT) can best be described as vague. Higher prices of the alternatives to combustible smoking are a major hurdle preventing their use for smoking cessation [7].

However, around the world, and particularly in Pakistan, there is a lack of smoking cessation program and nicotine awareness. Though nicotine is extremely addictive, other compounds in tobacco or tobacco smoke are responsible for the majority of illnesses [8]. Minimal evidence establishes nicotine's causative linkages to cancer and cardiovascular illness, and with regard to COPD, there is an inadequate data. Still, many believe nicotine causes smoking-related health problems such as cancer [9, 10]. These misunderstandings are not limited to the public. In one study, 60% of public health practitioners, such as nurses, mistook nicotine for a hazard [11].

According to a meta-analysis [12], health practitioner interventions had a substantial, albeit moderate, effect on smoking cessation when compared to normal care. The lung health study tracked 3320 NRT (nicotine gum) users for 7.5 years and discovered that smoking and NRT were not a significantpredictor of cancer [13]. The research team discovered that using nicotine gum was not linked to an increased risk of cardiovascular hospitalizations or fatalities following a five-year follow-up period [14]. A meta-analysis of the cardiovascular consequences of smoking cessation pharmacotherapies looked at 21 randomized controlled trials of NRTs and discovered an increased risk of all types of cardiovascular disease [15].

Nicotine awareness is lacking in the population and public health practitioners. Most of the quitting efforts are unsuccessful because smokers are becoming addicted to nicotine. Harm reduction is a public health approach that aims to lessen the harm caused by certain activities such as drug use. Modifying restrictions and prohibitions, empowering individuals with correct information, and promoting alternatives and the replacement of lower risk pharmaceuticals are some of such strategies [16]. However, in order to achieve effective smoking cessation, nicotine knowledge is crucial and vital. The purpose of this research is to determine the degree of nicotine knowledge among public health practitioners in Pakistan.

Section 2 includes research materials and procedures about the study region, data, sampling, instrument usage, and statistical framework.  Section 3 contains the findings, followed by discussion in Section 4.  Section 5 contains recommendations.

## 2. Materials and Methods

### 2.1. Study Area

This study investigates public health practitioners' knowledge of harm reduction and nicotine in Pakistan. This baseline research has been conducted in the twin-city districts of Islamabad and Rawalpindi (Figure 1). Islamabad is Pakistan's capital city, with a population of around two million.

Known as the garrison city, Rawalpindi is one of the largest districts in the Punjab province, with a population of 2.09 million. Islamabad is a higher and middle-income region, while Rawalpindi is a higher, middle, and low income region.

### 2.2. Data

Using primary survey data of 350 public health practitioners, a cross-sectional survey of public and private clinics and hospitals in Islamabad and Rawalpindi was conducted in October-November 2021. However, three respondents were excluded from the analysis due to missing information.  Table 1 contains the details of the cross-sectional sample.

### 2.3. Sampling

In light of the survey's objectives, a sample of 350 health practitioners was deemed adequate for obtaining reliable population parameter estimates within acceptable reliability limits. This study has used a 95% level of confidence, a 5% margin of error, and a 1 value of design effect to estimate the sample size. To calculate the required sample size, the following formula has been used:

(1) n=4r1−rdeffc^2,=400,

where *n* is the required sample size, expressed as number of health professionals,

4 is a factor to achieve the 95% level of confidence,

*r* is the predicted or anticipated value of the indicator, expressed in the form of a proportion,

deff is the design effect for the indicator, and

*c* is the margin of error.

The sample size of 400 was adjusted with the target population of health professionals and 350 was estimated to be sufficient for generlization and to yield reliable analysis.

#### 2.3.1. Sample Selection

For the selection of individual respondents, multistage simple random sampling was used. In the first stage, all possible doctors from the study area (Islamabad and Rawalpindi) were listed from public and private hospitals along with personal clinics. In the second stage, the required number of 350 responders was drawn at random from a pre-existing list of potential doctors.

### 2.4. Survey Instrument

This study has used structured questionnaire to collect information related to health professionals' knowledge of nicotine and tobacco products' health risk along with harm reduction products such as e-cigarettes, NRT, and non-NRT oral medications [17]. The questionnaire included precise definitions of all key concepts in order to allow the interviewer to refer to the definition during the interview. In addition, the questionnaire with instructional comments was translated into local language—Urdu. All questions were checked carefully to ensure they are not leading, or otherwise, likely to induce the respondent to give biased responses. Data was collected on android-based census and survey processing system (CSpro) application. Ensuring security and data consistency, android-based tablet devices were linked with a local server. The application had the provision of saving all collected data to safeguard against data loss during the synchronization process.

### 2.5. Content Validity

The field data automatically stored in the android-based CSpro application was cleaned to reduce the risk of measurement error. With Cronbach's alpha, the internal consistency of questions loaded onto the same factors such as nicotine's contribution to diseases and health risk scores for smoking products and components was assessed. Investigation of validity is based on the Principal Component Analysis (PCA).

### 2.6. Statistical Analysis

For statistical analysis, nonparametric tests, which included descriptive and inferential analyses, were conducted. The Kolmogorov-Smirnov test confirmed the underlying data had non-normal distributions. The median and range values describe continuous variables, while number and percentage values describe categorical variables. Differences between medians were assessed with Mann–Whitney U tests for the group analysis, and the Kruskal-Wallis H tests for more than two groups. Categorical variables were assessed with chi-square and Fisher's exact tests. All statistical tests were two-tailed, and the differences between groups considered statistically significant level were observed at 1%, 5%, and 10% of the *p* values. For statistical data analysis, Stata v15.1 has been used.

## 3. Results

The two subsections describe the descriptive and inferential analysis. The descriptive analysis identifies participants' characteristics in relation to nicotine-related health risks, tobacco products and components, and tobacco harm reduction (THR) products. Inferential analysis based on nonparametric techniques shows relationship between respondents' characteristics and the health risk of nicotine, tobacco products and components, and THR products.

### 3.1. Descriptive Analysis

Table 2 shows the characteristics of the respondents. In the twin cities of Rawalpindi and Islamabad, 347 doctors—240 male and 107 female—were interviewed. The majority of doctors worked in public hospitals (76%), followed by 16% in private hospitals, and 7% managed their own clinics. The majority of doctors (84%) did not get any particular training on smoking cessation. In Pakistan's tobacco control initiatives, lack of smoking cessation facilities is seen as a weak link. Furthermore, evidence shows smoking cessation is not high on the priority of doctors in the twin cities.

Doctors with wide range of specialties were interviewed. Half of them (49%) were general practitioners, followed by specialists (cardiologists, oncologists, pulmonologists, and neurologists) (28.5%), and family medicine (22.5%), respectively. Most doctors knew about cigarettes (98.9%), electronic cigarettes (79.5%), NRT (72.9%), and non-NRT (52.2%). However, not many (7.5%) knew about snus, an oral smokeless tobacco product.

Health professionals seem to be divided on the health risk of electronic cigarettes. Currently, the use of vaping products is limited in Pakistan. Legally imported, vaping products' outlets are in the upscale localities of major cities such as Karachi, Lahore, Islamabad, and Rawalpindi. Additionally, the perception of health professionals that the health risk of electronic cigarettes and smoking are equal may be influenced by their portrayal in the mainstream media globally and in Pakistan. It is clear that the health professionals' knowledge and perception about health risk of smoking alternatives needs clarity (Figures 2–3).

Health risk of smoking components, presented in Figure 4, shows a little more than half of doctors (56.2%) identified carbon monoxide as the most risky component, followed by tar (48.1%), tobacco (44.4%), and inhaled smoke (39.4%). It is interesting to note doctors saw nicotine as least risky component (29.9%). However, it is important to highlight mostly doctors believe nicotine causes cancer, cardiovascular disease, birth effects, and COPD. An overwhelming majority of doctors mistakenly believes nicotine is carcinogenic. More than two-thirds of doctors (70%) strongly agreed and 17.9% somewhat agreed with the statement that nicotine causes cancer. Almost 80% doctors strongly agreed with the statement that nicotine causes cardiovascular disease. However, 61.7% doctors correctly pointed out nicotine can cause birth defects while 81.6% held it responsible for COPD (Table 3).

Currently, doctors do not see electronic cigarettes as an alternative to reducing the risk of combustible smoking or as a product to help in quitting smoking (Table 4). A little more than one-fifth of doctors did not know about the electronic cigarettes. Overall doctors are divided on the safety of electronic cigarettes compared to tobacco; one-third thought electronic cigarettes were safer while 41.4% think otherwise, and one-fourth did not have any opinion in this regard. Almost half of the doctors (49%) did not see electronic cigarettes as effective in quitting smoking, and two-third would not recommend them as a cessation aid. Similarly, doctors (65.4%) thought electronic cigarettes should be prohibited.

### 3.2. Inferential Analysis

The PCA has been applied on variables vis-à-vis health risk scores for smoking products and components—combustible cigarettes, electronic cigarettes, snus, NRT, non-NRT, oral medications, nicotine, inhaled smoke, carbon monoxide, tobacco, and tobacco residue—in order to check the content validity of the survey instrument. PCA, a simple method for extracting relevant information from confusing datasets, has become a standard tool in data analysis in a variety of fields. It reduces a complicated dataset to a lower dimension, revealing hidden and simpler patterns. The principal components are new variables formed by linearly combining or mixing the original variables [7, 18, 19].

PCA attempts to pack as much information into the first component as possible and as little information into the second, and so on.  Table 5 depicts components that contributed to the data fluctuation. The first four components accounted for 88% of the total variation, along with multiple eigenvalues. The first component accounted for 44% of the total, followed by the second (21%), third (13%), and fourth (11%) components, and so on. Further, for values greater than one, eigenvalue represents the component's variance and is considered critical. The total number of variables is equal to the sum of all variables' values. The difference is the size of one component's eigenvalue compared to the next component's eigenvalue.

In an analysis, a scree plot is a line showing the eigenvalues of factors or major components. In an exploratory factor analysis, the scree plot identifies the number of factors to maintain or the number of principal components to keep in a PCA.  Figure 5 explains the first four components with maximum eigenvalues.

On a 10-point Likert-type scale ranging from 1 (low risk) to 10 (high risk), public health practitioners were asked to rate the perceived danger of smoking products and components in terms of health risk.  Table 6 shows the perceived risk (health scores) of e-cigarettes, snus, NRT, and non-NRT oral medications. Cigarettes had a median health risk score of 9, followed by electronic cigarettes and snus 7, NRT 5, and non-NRT with a score of 4. Further, nicotine health risk rating for each smoking component was less compared to tobacco, carbon monoxide, and tobacco residue (tar).

Tables 7 and 8 show the results of a cross analysis of tobacco products and components with respondent characteristics such as gender and smoking cessation training. There were no significant differences in perceived health risk scores for smoking products and components between male and female doctors, except for cigarettes, NRT, and nicotine where male doctors declared a lower risk. Smoking components such as inhaled smoke, carbon monoxide, tobacco, and tar had higher health risk rankings for male and female respondents. Surprisingly, there were statistically significant variations in perceived health risk ratings for smoking products and components, such as snus and NRT, between physicians who received and those who did not get any specific smoking cessation training. However, no statistically significant difference in perceived health risk ratings between physicians who received and those who did not get any specific smoking cessation training for nicotine at the 5% *p* value threshold. However, at the 10% *p* value threshold, it is statistically significant. Those who did not get any special training on smoking cessation evaluated high health risk ratings for combustible tobacco, electronic cigarettes, and tar. For carbon monoxide, tobacco and tar, there was no significant difference between the health professionals in terms of getting training, or otherwise, on smoking cessation.

There were also no statistically significant variations in perceived health risk rankings for smoking products between smokers (current and former) and nonsmoker doctors (Table 9). Respondents also expressed opinion on how significant nicotine is in the development of certain disorders. However, there was a statistically significant difference in perceived health risk for smoking components such as nicotine and carbon monoxide. Doctors who smoked (both current and former) did report less health hazards for nicotine than doctors who never smoked.

The score difference for smoking products and components between settings of practices (public, private, or own clinic) shows no significant differences. The average health risk rating of tobacco products, NRT, and non-NRT oral drugs was shown to be lower in public and private hospital doctors compared to other facility centers, but no statistical difference was detected (*p* = 0.20 and 0.37). When compared to tobacco and harm reduction products, the cross analysis of public health practitioners perception demonstrates that NRT and non-NRT oral drugs are rated less harmful to health. The average health risk rating of tobacco is higher than that of NRT and non-NRT cigarettes. Additionally, the public health practitioners rated higher health risk score for tobacco components such as nicotine, inhaled smoke, carbon monoxide, tobacco, and tar (Table 10).

The difference in score for smoking products and components between doctors' specialties shows no significant differences, except for cigarettes and NRT as products at 5% and 10% of *p* values, respectively. However, statistical difference has been observed in nicotine, inhaled smoke, and tobacco components at 1% and 10% of the *p* values. Family medicine specialists and general practitioners have demonstrated that the health risk score of products including NRT, non-NRT, and oral medications are lower. When compared to tobacco and e-cigarettes, the cross analysis of public health practitioner's perception demonstrates NRT and non-NRT oral drugs are less harmful to health. The average health risk rating of tobacco and electronic cigarettes is higher than that of NRT and non-NRT product. Specialists flagged a higher health risk score for tobacco components such as carbon monoxide, tobacco, and tar (Table 11).

Table 12 shows the health dangers of nicotine enlisted by doctors—smokers (current and former) and nonsmokers. The majority of nonsmoker doctors strongly agreed with the statement linking nicotine to cancer (72.2%), cardiovascular disease (81%), birth defects (63.2%), and COPD (83.5%). The smokers and nonsmoker doctors' perception regarding nicotine causing cancer and COPD is statistically significant.

The differences between male and female's perceptions regarding nicotine causing cancer, birth defects, and COPD were found to be significant. Majority of female doctors strongly believed nicotine causes cancer (77.6%), cardiovascular disease (84%), birth defects (70%), and COPD (90.7%). The difference is more pronounced over nicotine becoming one of the reasons for birth defect and COPD (Table 13).

Majority of doctors who had specific smoking cessation training strongly agreed that nicotine contributed to cancer (73.2%), cardiovascular disease (82.1%), birth defects (64.3%) and COPD (89.3%), respectively. Similarly, doctors with no specific smoking cessation training also strongly agreed that nicotine contributed to cancer (69.4%), cardiovascular disease (79.4%), birth defects (61.2%), and COPD (80.1%) (Table 14).

Similarly, there is no significant difference on the contribution of nicotine to diseases in terms of where the doctors worked—in public or private hospitals or managed their own clinics, except for the COPD. Only 8.7%, 4.5%, 9.4%, and 6.4% doctors working in public hospital doctors strongly disagree with the statements that nicotine causes cancer, cardiovascular disease, and birth abnormalities. Public and private hospitals or their own clinics statistically agreed on the 1% of *p* value that nicotine causes COPD. In contrast to public hospital doctors, health professionals working in private hospitals and their own clinics are less likely to believe that nicotine causes cancer, cardiovascular disease, and birth defects (Table 15).

The opinion on nicotine-related diseases in the context of specialties reveals significant differences regarding nicotine causes cancer and COPD at the 10% of the *p* value. Only 11% specialists of cardiology, pulmonary, oncology, and neurologist and 10.6% general practitioners strongly disagreed with the statement that nicotine causes cancer. Additionally, 8.2% general practitioners strongly disagreed that nicotine causes COPD. Most specialists believed nicotine causes cancer, cardiovascular, birth defects, and COPD (Table 16).

## 4. Discussion

To our knowledge, this is the first study on health professionals' perceptions regarding nicotine and other cigarette components in Pakistan. Doctors deemed NRT and non-NRT less harmful for health compared to combustible smoking. Health professionals seem to be divided on the health risk of electronic cigarettes. It may be because the use of electronic cigarettes in Pakistan is still limited. Additionally, the perception of health professionals that the health risk of electronic cigarettes and smoking are equal may be influenced by their portrayal in mainstream media globally and in Pakistan. It is clear the health professionals' knowledge and perception concerning health risk of smoking alternatives needs clarity. Several studies have found switching to electronic cigarettes leads to improved health. According to a research in the United States, based on the health information national trends survey, 51% of those who were aware of electronic cigarettes felt they were less risky than cigarettes [17]. A recent study that examined 72 eligible research papers to determine risk perceptions, including general harmfulness and specific health risks of electronic cigarettes, reported that adult vapers and adult smokers identified health advantages and good experiences with the electronic cigarette usage. Dual users and nonusers found no health advantages or good experiences. However, they did highlight some benefits for vapers in terms of desire reduction and safety [20]. The study emphasises the need for increased participation of health experts in the discussion of smoking prevalence and the potential contribution of THR to Pakistan's tobacco control efforts. At present, it seems that the tobacco use and its effects on health is not a pressing issue for health professionals.

When doctors were asked to rate the risk of components of combustible smoking, most termed carbon monoxide as the most dangerous, followed by tar, tobacco, and inhaled smoke (Figure 4). Besides nicotine, the cigarette produces more than 6,000 chemical particles, including nitrogen, carbon monoxide, and tar. These substances pose the greatest risks to health [21]. Studies show smoking kills millions of people worldwide every year. There are many different diseases, like those affecting the heart, lungs, mouth, stomach, and brain [22]. Moreover, smoking affects male and female fertility, sperm count, mobility, and increase the probability of miscarriage [23]. A recent study shows smoking is the leading cause of coronary heart disease, which affects people of all ages [24]. Most research indicates smokers have their own beliefs and presumptions. Most tobacco or cigarette users thought smoking helped them cope with their anxiety, stress, and depression [25]. According to certain studies, smokers puff cigarettes to reduce negative emotions and prevent unfavorable emotional disorders [26]. The relationship between smoking and psychological issues such as depression, stress, and anxiety is strong [27].

When it comes to the safety of electronic cigarettes compared to tobacco, doctors are divided. One-third termed them safer, while the remaining one-fourth were undecided. Nearly half of doctors believe electronic cigarettes are ineffective in helping smokers quit smoking. Two-thirds would not recommend them as a cessation aid (Table 3 and 4). When the doctors were asked to grade the products of combustible smoking in terms of risk, non-NRT and NRT were termed as least risky for health. However, a considerable number of doctors did not know about NRT health risk compared to combustible smoking. They also thought the risk of modified-risk tobacco products is lower than smoking (Table 6). In 1976, Michael Russell, who is considered the father of THR, said: “People smoke for the nicotine, but they die from the tar.” One of the first researchers to identify nicotine as the primary reason smokers become addicted, Russell was an early advocate of NRT. Among other proposals, Russell promoted low and medium nicotine and low tar cigarettes [28]. Tar paralyzes and can eventually kill cilia in the airways and when damaged, the toxins in tar can travel deeper into the lungs. Some of these toxins are released when one exhales or are coughed back out, but some settle and stay in lungs. Eventually, this can lead to lung disease and conditions such as emphysema, bronchitis, and lung cancer [29].

For both male and female doctors, smoking components such as inhaled smoke, carbon monoxide, tobacco, and tar had greater health risk rankings (Table 11). It is predetermined that combustible smoking is harmful to one's health, and new well-established information, action, and strategies can accomplish population-level benefits and avert the premature deaths of people globally. Product innovation, as well as tobacco/nicotine biobehavioral, epidemiological, and public health sciences show that low nitrosamine smokeless tobacco and alternative nicotine delivery systems (ANDS) cause far less damage than cigarettes [30].

When it came to the perceived health concerns of snus, NRT, and non-NRT, there was no significant difference between doctors who smoked and those who never smoked. For nicotine and carbon monoxide, there was statistically significant change in perceived health risk estimates (Table 9). The physicians need to be better informed about the fact that the primary risk of nicotine in tobacco products is addiction/dependence, but other carcinogens and chemicals, particularly those created by combustion, are the primary source of risk for tobacco-related illnesses [8].

The use of NRT and non-NRT oral medications was found to be lower in family medicine and general practice specialists. In terms of gender, the majority of female doctors feel nicotine plays a role in cancer, cardiovascular disease, birth defects, and COPD. When it came to doctors' attending smoking cessation training, the vast majority of those who did not agree that nicotine played a role in cancer, cardiovascular illness, birth defects, and COPD (Table 8). From the perspective of workplace—public or private hospital or own clinic—there was no substantial difference in opinion on nicotine-related disorders. However, the difference is evident when it comes to specializations. Majority of specialists thought nicotine was linked to cancer, cardiovascular disease, birth abnormalities, and COPD.

While it's possible that some doctors may have misinterpreted the question (for example, considering nicotine harmful rather than combustible tobacco), the findings are consistent with prior research on nicotine misperceptions [9, 10]. The Food and Drug Administration (FDA) proposed a nicotine-centered framework in 2017, which includes reducing nicotine content in cigarettes to nonaddictive levels while encouraging safer forms of nicotine use for harm reduction (e.g., smokeless tobacco) or cessation and correcting misconceptions. Reducing the addictiveness of cigarettes could make it easier for addicted smokers to stop and keep those who are just starting out, especially young people, from becoming regular smokers [31]. Additionally, misconceptions about nicotine can be easily corrected with short communication interventions[31–35].

## 5. Conclusions

Physicians in Pakistan have misconceptions about nicotine and THR. Majority links nicotine to cancer, cardiovascular disease, birth abnormalities, and COPD. They are also divided over effectiveness of smoking alternatives. The doctors' opinion about the nicotine-related diseases were imprecise. Physicians need to be better informed that the primary risk of nicotine in tobacco products is addiction/dependence. Other carcinogens and chemicals, particularly those created by combustion, are the primary source of risk for tobacco-related illnesses. Reducing the addictiveness of cigarettes could make it easier for smokers to stop and keep those who are just starting out, especially young people, from becoming regular smokers. Misconceptions about nicotine can be easily corrected with short communication interventions. A smoke-free Pakistan is possible in the near future. The first step in this direction can be broadening the horizon of the tobacco control efforts. The implementation of comprehensive tobacco control programs can lead to decrease in smoking prevalence and make THR the central plank of efforts for a smoke-free future. Effective cessation services should be accessible and affordable. Smokers' views should be heard, and THR should be part of the national tobacco control policy and innovative THR products should be sensibly regulated.

## Figures and Tables

**Figure 1:** Study Area.

**Figure 2:** Health professional perception about health risk of smoking products.

**Figure 3:** Health professional perception about health risk of smoking.

**Figure 4:** Health professional perception about health risk of smoking components.

**Figure 5:** Scree plot of the eigenvalues.

**Table 1:** Study sample.

District	%	*n*
Islamabad	58	201
Rawalpindi	42	146
Total	100	347

**Table 2:** Respondent characteristics.

Respondent characteristics		*n* (%)
Gender	Male	240 (69.0)
	Female	107 (31.0)

Setting of practice	Public hospitals	265 (76.0)
	Private hospitals	56 (16.0)
	Personal clinic	26 (7.0)

Specific training in smoking cessation	Yes	56 (16.0)
	No	291 (84.0)

Doctor's specialty	Specialist	99 (28.5)
	Family medicine	78 (22.5)
	General practitioner	170 (49.0)

Are you familiar with these products		

Tobacco cigarettes	Yes	343 (98.9)

Snus	Yes	26 (7.5)

Electronic cigarettes	Yes	276 (79.5)

NRT	Yes	253 (72.9)

Non-NRT	Yes	181 (52.2)

**Table 3:** Perception about nicotine.

	Strongly agree	Somewhat agree	Somewhat disagree	Strongly disagree	Do not know
Nicotine causes cancer	70.0	17.9	1.4	9.8	0.9
Nicotine causes cardiovascular disease	79.8	12.7	1.4	4.6	1.4
Nicotine causes birth defects	61.7	21.6	4.0	8.1	4.6
Nicotine causes COPD	81.6	9.2	1.7	6.6	0.9

**Table 4:** Perception about e-cigarettes.

	Yes	No	Do not know
Electronic cigarettes can generate addiction	68.0	8.9	23.1
Electronic cigarettes are more expensive than normal tobacco	72.9	2.9	24.2
Electronic cigarettes are safer than tobacco	33.1	41.8	25.1
Electronic cigarettes are effective devices for smoking cessation	26.5	49.0	24.5
Would you recommend electronic cigarette as smoking cessation aid?	11.8	66.3	21.9
Do you think that medical community and healthcare workers should take a position in favour of the electronic cigarettes?	13.5	63.7	22.8
Do you think that electronic cigarettes should be prohibited?	65.4	11.8	22.8

**Table 5:** PCA Analysis.

Component	Eigenvalue	Difference	Proportion	Cumulative
1	4.37	2.29	0.44	0.44
2	2.08	0.80	0.21	0.64
3	1.28	0.21	0.13	0.77
4	1.07	0.50	0.11	0.88
5	0.57	0.16	0.06	0.94
6	0.41	0.26	0.04	0.98
7	0.15	0.09	0.01	0.99
8	0.06	0.04	0.01	1.00
9	0.02	0.01	0.00	1.00
10	0.00	.	0.00	1.00

**Table 6:** Health risk scores for smoking products and components.

Product (*n*)	Median and range
Tobacco cigarettes (*n* = 341)	9 (1-10)
Electronic cigarettes (*n* = 276)	7 (2-10)
^∗^Snus (*n* = 26)	7 (1-10)
NRT (*n* = 251)	5 (1-10)
Non-NRT oral medications (*n* = 180)	4 (1-10)
*Component(*n*)*	
Nicotine (*n* = 345)	8 (1-10)
Inhaled smoke (*n* = 345)	9 (1-10)
Carbon monoxide (*n* = 345)	10 (1-10)
Tobacco (*n* = 345)	9 (1-10)
Tar (*n* = 345)	9 (1-10)

NRT, tar, tobacco residue, ^∗^health experts' knowledge of snus was quite low.

**Table 7:** Differences in score for smoking products and components between male and female health professionals.

Product (*n*)	Male (*n* = 240)	Female (*n* = 107)	
	Median and range	Median and range	*p* value
Tobacco cigarettes	9 (1-10)	9 (4-10)	0.04^∗∗^
Electronic cigarettes	7 (2-10)	8 (4-10)	0.25
Snus	7 (1-10)	7.5 (2-10)	0.13
NRT	4 (1-10)	5 (1-10)	0.03^∗∗^
Non-NRT oral medications	4 (1-10)	5 (1-10)	0.18
*Component(*n*)*			
Nicotine	7 (1-10)	9 (2-10)	0.00^∗^
Inhaled smoke	9 (1-10)	9 (3-10)	1.00
Carbon monoxide	10 (1-10)	10 (4-10)	0.19
Tobacco	9 (1-10)	9 (3-10)	0.69
Tar	9 (1-10)	9 (4-10)	0.67

^∗^at 1% of *p* value, ^∗∗^at 5% of *p* value, ^∗∗∗^at 10% of *p* value.

**Table 8:** Differences in score for smoking products and components between smoking cessation trained and nontrained health professionals.

Product (*n*)	Trained (*n* = 56)	Not-trained (*n* = 289)	
	Median and Range	Median and Range	*p* value
Tobacco cigarettes	10 (1-10)	9 (1-10)	0.35
Electronic cigarettes	8 (5-10)	7 (2-10)	0.25
Snus	8 (1-10)	7 (1-10)	0.02^∗∗^
NRT	5 (1-10)	4 (1-10)	0.02^∗∗^
Non-NRT oral medications	4 (1-10)	4 (1-10)	0.22
*Component(*n*)*			
Nicotine	8 (1-10)	8 (1-10)	0.07^∗∗∗^
Inhaled smoke	9 (3-10)	9 (1-10)	0.26
Carbon monoxide	9 (1-10)	10 (1-10)	0.32
Tobacco	9 (1-10)	9 (1-10)	0.22
Tar	10 (1-10)	9 (1-10)	0.14

^∗^at 1% of *p* value, ^∗∗^at 5% of *p* value, ^∗∗∗^at 10% of *p* value.

**Table 9:** Differences in score for smoking products and components between smokers and nonsmokers health professionals.

Product (*n*)	Smokers (current and former) (*n* = 56)	Never smokers (*n* = 291)	
	Median and range	Median and range	*p* value
Tobacco cigarettes	8 (1-10)	9 (3-10)	0.88
Electronic cigarettes	5 (5-7)	8 (2-10)	0.28
Snus	7 (1-10)	7 (1-10)	0.64
NRT	4 (1-10)	5 (1-10)	0.26
Non-NRT oral medications	4 (1-10)	4 (1-10)	0.93
*Component(*n*)*			
Nicotine	7 (1-10)	8 (1-10)	0.02∗∗
Inhaled smoke	9 (3-10)	9 (1-10)	0.90
Carbon monoxide	9.5 (1-10)	10 (1-10)	0.00∗
Tobacco	9 (1-10)	9 (1-10)	0.90
Tar	9 (1-10)	9 (1-10)	0.85

**Table 10:** Differences in score for smoking products and components between settings of practices.

Product (*n*)	Public hospital (*n* = 265)	Private hospital (*n* = 56)	Other facilities (*n* = 26)	
	Median and range	Median and range	Median and range	*P* value
Tobacco cigarettes	9 (1-10)	10 (3-10)	8.5 (6-10)	0.34
Electronic cigarettes	7 (2-10)	10 (5-10)	6 (6-6)	0.12
Snus	7 (1-10)	9 (2-10)	6 (4-10)	0.01^∗^
NRT	4 (1-10)	5 (1-10)	5 (1-10)	0.20
Non-NRT oral medications	4 (1-10)	4 (1-10)	5 (3-7)	0.37
*Component(*n*)*				
Nicotine	8 (1-10)	9 (3-10)	8 (1-10)	0.41
Inhaled smoke	9 (1-10)	9 (3-10)	8 (5-10)	0.16
Carbon monoxide	10 (1-10)	8 (1-10)	9.5 (5-10)	0.01^∗^
Tobacco	10 (1-10)	8 (1-10)	9 (4-10)	0.05^∗∗^
Tar	9 (1-10)	9 (3-10)	8 (4-10)	0.26

^∗^at 1% of *p* value, ^∗∗^at 5% of *p* value, ^∗∗∗^at 10% of *p* value.

**Table 11:** Differences in score for smoking products and components between doctor's specialties.

Product (*n*)	Specialist (*n* = 99)	Family medicine (*n* = 78)	General practitioners (*n* = 170)	
	Median and range	Median and range	Median and range	*p* value
Tobacco cigarettes	8 (1-10)	9.5 (3-10)	9 (1-10)	0.02^∗∗^
Electronic cigarettes	8 (6-10)	6 (4-10)	7 (1-10)	0.34
Snus	6 (1-10)	7 (2-10)	7 (1-10)	0.31
NRT	4 (1-10)	5 (1-10)	5 (1-10)	0.06^∗∗∗^
Non-NRT oral medications	4 (1-10)	5 (1-10)	4 (1-10)	0.10^∗∗∗^
*Component(*n*)*				
Nicotine	7 (1-10)	8 (1-10)	8 (1-10)	0.00^∗^
Inhaled smoke	8 (3-10)	9 (3-10)	9 (1-10)	0.07^∗∗∗^
Carbon monoxide	10 (1-10)	10 (1-10)	10 (1-10)	0.19
Tobacco	10 (1-10)	9 (3-10)	9 (1-10)	0.08^∗∗∗^
TAR	9 (1-10)	9 (3-10)	9 (3-10)	0.66

^∗^at 1% of *p* value, ^∗∗^at 5% of *p* value, ^∗∗∗^at 10% of *p* value.

**Table 12:** Contribution of nicotine to diseases: differences between smoker and nonsmoker practitioners.

Disease	Smokers (current and former) (*n* = 56)	Never smokers (*n* = 288)	*p*
	*n* (%)	*n* (%)	
*Nicotine causes cancer*			
Strongly agree	33 (58.9)	210 (72.2)	0.01^∗^
Somewhat agree	10 (17.9)	52 (17.9)	
Somewhat disagree	1 (1.8)	4 (1.4)	
Strongly disagree	12 (21.4)	22 (7.6)	
Do not know	0 (0)	3 (1.0)	
*Nicotine causes cardiovascular*			
Strongly agree	41 (73.2)	236 (81.1)	0.13
Somewhat agree	7 (12.5)	37 (12.7)	
Somewhat disagree	1 (1.78)	4 (1.4)	
Strongly disagree	6 (10.7)	10 (3.4)	
Do not know	1 (1.8)	4 (1.4)	
*Nicotine causes birth defects*			
Strongly agree	30 (53.6)	184 (63.2)	0.14
Somewhat agree	14 (25.0)	61 (21.0)	
Somewhat disagree	1 (1.8)	13 (4.5)	
Strongly disagree	8 (14.3)	20 (6.9)	
Do not know	3 (5.4)	13 (4.5)	
*Nicotine causes COPD*			
Strongly agree	40 (71.4)	243 (83.5)	0.01^∗^
Somewhat agree	5 (8.9)	27 (9.3)	
Somewhat disagree	2 (3.6)	4 (1.4)	
Strongly disagree	9 (16.1)	14 (4.8)	
Do not know	0 (0)	3 (1.0)	

^∗^at 1% of *p* value, ^∗∗^at 5% of *p* value, ^∗∗∗^at 10% of *p* value.

**Table 13:** Contribution of nicotine to diseases: differences between male and female practitioners.

Disease	Male (*n* = 240)	Female (*n* = 107)	*p*
	*n* (%)	*n* (%)	
*Nicotine causes cancer*			
Strongly agree	160 (66.7)	83 (77.6)	0.02^∗∗^
Somewhat agree	44 (18.3)	18 (16.8)	
Somewhat disagree	3 (1.3)	2 (1.9)	
Strongly disagree	31 (12.9)	3 (2.8)	
Do not know	2 (0.8)	1 (0.9)	
*Nicotine causes cardiovascular*			
Strongly agree	187 (77.9)	90 (84.1)	0.12
Somewhat agree	29 (12.1)	15 (14)	
Somewhat disagree	4 (1.7)	1 (0.9)	
Strongly disagree	16 (6.7)	0 (0)	
Do not know	4 (1.7)	1 (0.9)	
*Nicotine causes birth defects*			
Strongly agree	139 (57.9)	75 (70.1)	0.03^∗∗^
Somewhat agree	57 (23.8)	18 (16.8)	
Somewhat disagree	8 (3.3)	6 (5.6)	
Strongly disagree	23 (9.6)	5 (4.7)	
Do not know	13 (5.4)	3 (2.8)	
*Nicotine causes COPD*			
Strongly agree	186 (77.5)	97 (90.7)	0.00^∗^
Somewhat agree	23 (9.6)	9 (8.4)	
Somewhat disagree	5 (2.1)	1 (0.9)	
Strongly disagree	23 (9.6)	0 (0)	
Do not know	3 (1.3)	0 (0)	

^∗^at 1% of *p* value, ^∗∗^at 5% of *p* value, ^∗∗∗^at 10% of *p* value.

**Table 14:** Contribution of nicotine to diseases: differences between smoking cessation trained and non-trained practitioners.

Disease	Yes (*n* = 56)	No (*n* = 291)	*p*
	*n* (%)	*n* (%)	
*Nicotine causes cancer*			
Strongly agree	41 (73.2)	202 (69.4)	0.30
Somewhat agree	14 (25)	48 (16.5)	
Somewhat disagree	0 (0)	5 (1.7)	
Strongly disagree	1 (1.8)	33 (11.3)	
Do not know	0 (0)	3 (1)	
*Nicotine causes cardiovascular*			
Strongly agree	46 (82.1)	231 (79.4)	0.59
Somewhat agree	7 (12.5)	37 (12.7)	
Somewhat disagree	1 (1.8)	4 (1.4)	
Strongly disagree	2 (3.6)	14 (4.8)	
Do not know	0 (0)	5 (1.7)	
*Nicotine causes birth defects*			
Strongly agree	36 (64.3)	178 (61.2)	0.48
Somewhat agree	14 (25)	61 (21)	
Somewhat disagree	1 (1.8)	13 (4.5)	
Strongly disagree	3 (5.4)	25 (8.6)	
Do not know	2 (3.6)	14 (4.8)	
*Nicotine causes COPD*			
Strongly agree	50 (89.3)	233 (80.1)	0.10^∗∗∗^
Somewhat agree	3 (5.4)	29 (10)	
Somewhat disagree	1 (1.8)	5 (1.7)	
Strongly disagree	2 (3.6)	21 (7.2)	
Do not know	0 (0)	3 (1)	

^∗^at 1% of *p* value, ^∗∗^at 5% of *p* value, ^∗∗∗^at 10% of *p* value.

**Table 15:** Contribution of nicotine to diseases: differences between settings of practitioners.

Disease	Public hospital (*n* = 265)	Private hospital (*n* = 56)	Other facilities (*n* = 26)	*p*
	*n* (%)	*n* (%)	*n* (%)	
*Nicotine causes cancer*				
Strongly agree	189 (71.3)	37 (66.1)	17 (65.4)	0.43
Somewhat agree	49 (18.5)	9 (16.1)	4 (15.4)	
Somewhat disagree	4 (1.5)	0 (0)	1 (3.8)	
Strongly disagree	23 (8.7)	7 (12.5)	4 (15.4)	
Do not know	0 (0)	3 (5.4)	0 (0)	
*Nicotine causes cardiovascular*				
Strongly agree	217 (81.9)	40 (71.4)	20 (76.9)	0.15
Somewhat agree	32 (12.1)	9 (16.1)	3 (11.5)	
Somewhat disagree	3 (1.1)	1 (1.8)	1 (3.8)	
Strongly disagree	12 (4.5)	2 (3.6)	2 (7.7)	
Do not know	1 (0.4)	4 (7.1)	0 (0)	
*Nicotine causes birth defects*				
Strongly agree	168 (63.4)	32 (57.1)	14 (53.8)	0.70
Somewhat agree	52 (19.6)	15 (26.8)	8 (30.8)	
Somewhat disagree	8 (3)	4 (7.1)	2 (7.7)	
Strongly disagree	25 (9.4)	2 (3.6)	1 (3.8)	
Do not know	12 (4.5)	3 (5.4)	1 (3.8)	
*Nicotine causes COPD*				
Strongly agree	224 (84.5)	37 (66.1)	22 (84.6)	0.01^∗^
Somewhat agree	19 (7.2)	11 (19.6)	2 (7.7)	
Somewhat disagree	5 (1.9)	0 (0)	1 (3.8)	
Strongly disagree	17 (6.4)	5 (8.9)	1 (3.8)	
Do not know	0 (0)	3 (5.4)	0 (0)	

^∗^at 1% of *p*value, ^∗∗^at 5% of *p* value, ^∗∗∗^at 10% of *p* value.

**Table 16:** Contribution of nicotine to diseases: differences between practitioners specialties.

Disease	Specialist (*n* = 99)	Family medicine (*n* = 78)	General practitioners (*n* = 170)	*p*
	*n* (%)	*n* (%)	*n* (%)	
*Nicotine causes cancer*				
Strongly agree	73 (73.7)	61 (78.2)	109 (64.1)	0.06^∗∗^
Somewhat agree	13 (13.1)	12 (15.4)	37 (21.8)	
Somewhat disagree	1 (1)	0 (0)	4 (2.4)	
Strongly disagree	11 (11.1)	5 (6.4)	18 (10.6)	
Do not know	1 (1.0)	0 (0)	2 (1.2)	
*Nicotine causes cardiovascular*				
Strongly agree	82 (82.8)	65 (83.3)	130 (76.5)	0.34
Somewhat agree	10 (10.1)	8 (10.3)	26 (15.3)	
Somewhat disagree	0 (0)	2 (2.6)	3 (1.8)	
Strongly disagree	6 (6.1)	2 (2.6)	8 (4.7)	
Do not know	1 (1.0)	1 (1.3)	3 (1.8)	
*Nicotine causes birth defects*				
Strongly agree	60 (60.6)	51 (65.4)	103 (60.6)	0.50
Somewhat agree	23 (23.2)	19 (24.4)	33 (19.4)	
Somewhat disagree	0 (0)	3 (3.8)	11 (6.5)	
Strongly disagree	7 (7.1)	4 (5.1)	17 (10)	
Do not know	9 (9.1)	1 (1.3)	6 (3.5)	
*Nicotine causes COPD*				
Strongly agree	82 (82.8)	69 (88.5)	132 (77.6)	0.09^∗∗∗^
Somewhat agree	9 (9.1)	7 (9)	16 (9.4)	
Somewhat disagree	0 (0)	0 (0)	6 (3.5)	
Strongly disagree	7 (7.1)	2 (2.6)	14 (8.2)	
Do not know	1 (1.0)	0 (0)	2 (1.2)	

^∗^at 1% of *p* value, ^∗∗^at 5% of *p* value, ^∗∗∗^at 10% of *p* value.

## Data Availability

All relevant data are within the paper and an additional data can be provided on demand.
